# Therapeutic Effect of Astragali Radix Extract Injection Combined with Bone Marrow Mesenchymal Stem Cells in Bleomycin-Induced Pulmonary Fibrotic Rats

**DOI:** 10.1155/2022/4933255

**Published:** 2022-06-13

**Authors:** Quanyu Du, Xuanyu Wu, Liping An, Rui Zhou, Xiang Xiao, Cheng Wu, Fei Wang, Han Yang

**Affiliations:** ^1^Endocrine Department, Hospital of Chengdu University of Traditional Chinese Medicine, Chengdu 610072, China; ^2^Geriatrics Department, Hospital of Chengdu University of Traditional Chinese Medicine, Chengdu 610072, China; ^3^Department of Pathology, Hospital of Chengdu University of Traditional Chinese Medicine, Chengdu 610072, China

## Abstract

Pulmonary fibrosis is a serious disease for which effective drugs are unavailable. Here, we treated rat models of bleomycin (BLM)-induced pulmonary fibrosis with Astragali Radix extract injection (AI) combined with or without bone marrow mesenchymal stem cells (BMSCs). We injected rats intratracheally with BLM and transplanted BMSCs *via* tail vein injection 15 days later. We also intraperitoneally injected AI daily from days 15 to 28. Changes in lung pathology and function, as well as the levels of matrix metalloproteinases, collagen, C-X-C motif chemokine ligand 12 (CXCL12), and cluster of differentiation 90 (CD90) were assessed. The results revealed that compared with the BLM group, groups treated with ARE and BMSCs (alone or combined) reduced the expression levels of TGF-*β*1 and collagens I and III, ameliorated pathological lung fibrotic damage, and improved lung function. The expression levels of MMP-1, MMP-3, and MMP-9 were reduced by either AI or BMSCs alone, whereas those of MMP-3, MMP-9, TIMP-1, CXCL12, and CD90 were elevated by combined AI and BMSCs compared with the BLM group. Overall, these findings demonstrated that AI and BMSCs both can reduce damage caused by PF in rats and that AI altered the expression of chemokines and surface markers in BMSCs.

## 1. Introduction

Primary and secondary forms of pulmonary fibrosis (PF) are widespread global health concerns that are characterized by extracellular matrix deposition in the lung and destruction of the lung structure. The most severe form of PF is idiopathic PF (IPF), which is age-related, characterized by dyspnea and progressive deterioration of lung function, and often results in death within 3–5 years of diagnosis [1]. The incidence of PF has recently increased, and patients with novel coronavirus pneumonia, especially those who are critically ill, often have residual pulmonary fibrosis [2–4]. Pulmonary fibrosis is also associated with chronic obstructive pulmonary disease [5], diabetes mellitus [6], and other chronic diseases that reduce the quality of life (QOL) and survival of patients. However, the mechanism of PF is complex, and glucocorticoids and immunosuppressants, for example, do not improve fibrotic status [7, 8]. The search for effective and tolerable therapeutic strategies for treating PF is an urgent issue for investigators.

Traditional Chinese medicine (TCM) is widely used to help treat PF. Their therapeutic effects are associated with improving lung function and the QOL of patients [9, 10]. Drugs such as Astragalus [11] that tonify Qi are the most popular drug type of herbs for treating PF. Astragalus can regulate the immune function of patients with PF and reduce inflammation and collagen content in lung tissues [12, 13].

Mesenchymal stem cell (MSC) transplantation is a new approach to treating PF [14]. These cells can reduce the inflammatory response, promote epithelial repair, and reduce the deposition of pulmonary extracellular matrix in PF lung tissues through multidirectional differentiation, immune regulation, and paracrine functions [15]. Astragalus and its metabolites can promote the proliferation, differentiation, and migration of MSCs [16–18]. However, whether Astragalus and MSCs have synergistic effects against PF remains unclear. Here, we assessed the effects of Astragali Radix extract injection (AI) combined with BMSC transplantation in model rats with bleomycin (BLM)-induced PF and revealed its potential role and mechanism in treating PF (Figure 1).

## 2. Materials and Methods

### 2.1. Animals

Male-specific pathogen-free (SPF) neonatal Sprague-Dawley (SD) rats aged 14–20 days and male SPF adult SD rats (weight, 250 + 20 g) were obtained from Chengdu Dashuo Laboratory Animal Co. (Certificate No. SCXK2020-030). We extracted BMSCs from the neonatal rats and used the adult rats for experiments *in vivo*. Adult rats were housed at the Affiliated Hospital of Chengdu University of Traditional Chinese Medicine throughout the experimental period at 21°C–23°C and 50%–55% relative humidity under 12-hour light/dark photoperiods, with access to food and water *ad libitum*. The experimental procedures complied with international and national ethical regulations as with strict adherence to all animal welfare guidelines.

### 2.2. Drugs and Reagents

The following were obtained from the respective suppliers: pirfenidone (Cat. no. H20133376; Beijing Kantini Pharmaceutical Co., Ltd., Beijing, China), Astragali Radix injection (Cat. no. Z13020999; Shenwei Pharmaceutical Group Co., Ltd., Shijiazhuang, China), bleomycin (Cat. no. S121418; Selleck Chemicals LLC., Houston, TX, USA), animal total RNA extraction kit (Cat. no. RE-03014; Chengdu Fuji Biotechnology Co., Ltd. Chengdu, China), primers (Shanghai Bioengineering Co., Ltd., Shanghai, China), ELISA kits for tissue inhibitor matrix metalloproteinase 1 (TIMP-1), MMP-1, MMP-2, MMP-3, MMP-9, C-X-C motif chemokine ligand 12 (CXCL12), and Transforming Growth Factor 1 (TGF-*β*1) (Cat. nos. VYC8QH5NYN, 75VQXXRG5Q, 2L4FL9TRE6, W3B59JV1PK, 1H4I373DP9, L82R7TXILH, and YFJI5U2X3T1031, respectively; Wuhan Elite Biotechnology Co., Ltd., Wuhan, China), fluorescent-labeled sheep anti-mouse IgG (Cat. no. BA1031; Boster Biological Technology, Co., Ltd., Pleasanton, CA, USA), and cluster of differentiation 90 (CD90) antibody (Cat. no. ab33694; Abcam, Cambridge, UK).

### 2.3. Isolation, Culture, and Identification of Rat Bone Marrow Mesenchymal Stem Cells

Rat bone marrow mesenchymal stem cells were isolated and cultured as described [19]. Neonatal rats were sacrificed by cervical dislocation, immersed in 75% alcohol for 5 min, and fixed supine on a sterilized worktable. The femurs and tibias of the rats were aseptically isolated; then, bone marrow cavities were exposed. The bone marrow was repeatedly washed with Minimum Essential Medium alpha (MEM*α*) until it turned white. Bone marrow suspensions were filtered through a 200-mesh sieve and centrifuged at 1,200 rpm for 5 min, and then, the pellets were resuspended in MEM*α*. Suspensions were centrifuged with rat lymphocyte separation solution at 2,000 rpm for 20 min. Leukoplakia cells in the middle of centrifuge tubes were taken as BMSCs, and 2 × 10^6^ cells/mL were inoculated into dishes and cultured at 37°C under 5% CO_2_. The medium was changed every three days. Fully grown cells were transferred to the P2 generation for standby tests. The expression of CD90, a BMSC marker, was detected using immunofluorescence staining. Thereafter, BMSCs were fixed on slides with 4% paraformaldehyde. Nonspecific antigen binding was blocked with goat serum for 30 min, and then, the slides were incubated with CD90 primary antibody at 4°C overnight. The slides were immersed in PBST and incubated in darkness for 1 h with fluorescent-labeled sheep anti-mouse IgG. Thereafter, nuclei were stained with DAPI, and the slides were sealed and visualized using fluorescence microscopy images.

### 2.4. Model Preparation and Administration

Adult SD rats were acclimatized for one week and then randomly assigned to the following groups (*n* = 6 per group): sham-operated (Sham), bleomycin (BLM), IPF drug pirfenidone (PFD), bone marrow mesenchymal stem cells (BMSCs), AI alone (AI), and AI with BMSCs (AI + BMSC). Pulmonary fibrosis was modeled using BLM (5 mg/kg) delivered *via* an endotracheal drip to anesthetized rats after surgical exposure [20]. The rats in the sham group underwent the same surgical procedure but were injected with equal volumes of saline. Drugs were started 14 days after BLM injection. The BMSC and AI + BMSC groups were injected once through the caudal vein with 0.3 mL of BMSCs (2 × 10^6^/mL) and then treated with drugs. Both the AI + BMSC and AI groups were intraperitoneally injected with AI 10 mL/kg/day; the PFD group received 100 mg/kg/day of PFD by gavage; and the sham and BLM groups were intraperitoneally injected with the same dose of normal saline for 14 days. The rats were fasted for 8 h after the last administration, and lung function was examined in rats anesthetized with pentobarbital sodium (30 mg/kg). Blood was then sampled from the abdominal aorta, and lung tissues were removed. The left lungs were fixed in 4% paraformaldehyde, and the right lungs were frozen at −80°C.

### 2.5. Pulmonary Function Test

The rats were anesthetized with sodium pentobarbital and then intubated *via* tracheotomy. The lung function of the rats was measured using an AniRes2005 Animal Lung Function Analysis system (Beijing Beranbo Technology Co., Beijing, China). The rats were placed supine in a medium-sized body drawing box, then a ventilator was connected, and the box was closed. The breathing rate, breathing ratio, and pressure were 65/min, 20 : 10, and 30 cm H_2_O, respectively. We measured forced vital capacity (FVC) and dynamic lung compliance (CYDN) [21].

### 2.6. Enzyme-Linked Immunosorbent Assay (ELISA)

Frozen rat serum was thawed and analyzed using TIMP-1, MMP-1, MMP-2, MMP-3, MMP-9, CXCL12, and TGF-*β*1 ELISA kits as described by the manufacturer. Maximum absorption was measured at a wavelength of 450 nm, and protein contents were calculated from standard curves [22].

### 2.7. Fluorescence Quantitative Reverse Transcriptase-Polymerase Chain Reaction (RT-qPCR)

Total RNA was extracted from homogenates of thawed lung tissues stored at −80°C and quantified. Complementary DNA synthesized by reverse transcription served as the template for PCR amplification under conditions of 95°C for 10 min, followed by 40 cycles of 95°C for 10 s and 60°C for 30 s with the primers listed in Table 1. The internal standard was *β*-actin, and the relative expression levels of the target genes were calculated using the 2^−ΔΔCt^ method [23].

### 2.8. Histological Analysis

Lung tissues were fixed in 4% paraformaldehyde for 48 h, then paraffin-embedded, cut into 5-*μ*m sections, and stained with hematoxylin and eosin (HE) and Masson trichrome using a standard protocol as described by the manufacturer. The steps included dewaxing, staining, transparency, and sealing as described in the instructions. Areas of stained collagen fibers were quantified using ImageJ software; then, the collagen volume fraction (%) was calculated as the area of collagen fiber/area of total view [24].

### 2.9. Statistical Analysis

All data were statistically analyzed using GraphPad Prism v. 8.0 (GraphPad Software Inc., San Diego, CA, USA) and are expressed as means ± SD. Comparisons among multiple groups and data with normal distribution were analyzed using one-way ANOVA. Data without normal distribution were analyzed using the Kruskal–Wallis test. Values with *P* < 0.05 were considered statistically significant.

## 3. Results

### 3.1. Positive Expression of CD90, A Marker of Primary BMSCs

The ratio of BMSCs emitting red fluorescence indicating positive CD90 expression was >90% (Figure 2). This met the requirements for using the BMSCs for experimental PF treatment.

### 3.2. Astragali Radix Extract Injection Combined with BMSCs Reduced Impaired Lung Function and Pulmonary Fibrosis in BLM Rats

Lung function was measured 28 days after the BLM injection. The FVC (Figure 3(a)) and CYDN were significantly lower in the BLM than in the sham group (Figure 3(b)). Astragali Radix extract injection with or without BMSCs increased the FVC and CYDN in the BLM and positive control PFD group. The alveolar structure of rat lung tissues stained with HE was intact in the sham group (Figure 3(c)). In contrast, lung tissues were severely disrupted, with significantly thickened alveolar septa, some ruptured alveolar walls, and more inflammatory cells in some locations in the model (Figure 3(d)) compared with the sham group. Four groups were treated with drugs that repaired the damaged lung tissues to some extent compared with the model, and the alveolar structure was intact in most areas of the section, with alveolar septum thickening and inflammatory cell infiltration in a few areas. Figures 3(f)–3(h) show that the alveolar structures of the BMSC, AI + BMSC, and AI groups were typically more intact. Masson staining revealed no apparent areas of fiber staining in the sham group (Figure 3(i)), except around bronchi and blood vessels. Areas of blue staining around the bronchi and blood vessels were broader and darker in the BLM than in the sham group. All images in Figure 3 were acquired while avoiding the large bronchi and blood vessels. However, more areas were stained blue in the alveolar region in the BLM group (Figure 3(j)). Among the six sets of slices analyzed using ImageJ software, the ratio of the area of blue collagen staining to that of the total section was significantly higher in the BLM (Figure 3(o)), than in any other groups. The four groups treated with drugs (Figures 3(k)–3(n)) had more intact lung tissue, with improved alveolar septal thickening and collagen deposition, than the BLM group.

### 3.3. Regulated Expression of Transforming Growth Factor Beta 1 (TGF-*β*1), MMPs, and Their Inhibitors in BLM Rats

The expression level of TGF-*β*1 in the serum of BLM-induced rats was increased, and cell growth and differentiation were promoted. The expression levels of MMP-1, MMP-2, MMP-3, MMP-9, and their inhibitor TIMP-1 simultaneously increased. The mRNA levels of collagen I and collagen III, the main components of the extracellular matrix, were also increased in the lung tissues. Among the factors closely associated with the occurrence and development of PF, the expression levels of other proteins and genes (except MMP-2, TIMP-1, and collagen III) significantly differed between the BLM and sham groups. Both the AI and the BMSC groups had reduced expression levels of TGF-*β*1, MMP-1, MMP-3, MMP-9, TIMP-1, and collagens I and III compared with BLM. The difference was that in the AI + BMSC group, AI simultaneously promoted MMP-2, MMP-3, MMP-9, and TIMP-1 in the serum of BLM rats transplanted with BMSCs and the expression levels of MMPs and their inhibitors increased. Although these markers increased in the AI + BMSC group, collagen expression in lung tissues notably decreased (Figure 4).

### 3.4. Promotion of CXCL12, C-X-C Chemokine Receptor 4 (CXCR4), and CD90 Expression

C-X-C motif chemokine ligand 12 is an important chemokine that drives the migration of stem cells in specific directions, and CXCR4 is its receptor. Serum levels of CXCL12 and CD90, a surface marker for BMSCs in lung tissues, were reduced in the BLM compared with the sham group. The expression levels of CXCL12 and CD90 increased in the AI and BMSC groups. Significantly more CXCL12 and CD90 were expressed in the AI + BMSC than in the model group (Figure 5).

## 4. Discussion

Pulmonary fibrosis is a severe group of lung diseases characterized by the excessive proliferation of lung fibroblasts with massive extracellular matrix deposition and structural destruction of the lungs. It results from various interstitial lung diseases and can develop from acute and chronic lung injuries.

Traditional Chinese Medicine is a unique medical treatment for PF that functions *via* a multilevel and multitarget approach [25]. Pulmonary fibrosis from the viewpoint of TCM is associated with external Qi such as wind, cold, damp, and heat, causing lung damage. Various chronic diseases constantly deplete the body of positive Qi, leading to lung Qi deficiency and stagnant blood circulation. Phlegm, deficient Qi, and blood stasis are the pathological features of PF according to TCM. Therefore, supplementing Qi and activating blood circulation are core TCM treatments for PF.

Either TCM alone or combined with Western medicine benefits pulmonary function in patients with PF. It can improve the FEV1 as well as the diffusion capacity for carbon monoxide in the lungs. Chinese medicine can also improve the exercise ability of patients, increase the 6-min walking time, and reduce St. George respiratory questionnaire scores [26]. Chinese herbs for supplementing Qi and activating blood circulation combined with N-acetylcysteine or pirfenidone can regulate the FVC of patients with PF [27]. Danggui Buxue and Buyang Huanwu decoctions, as well as other classical prescriptions for supplementing Qi and activating blood circulation, are also protective in animal models of PF *in vivo.* These prescriptions inhibit pulmonary inflammation, collagen deposition, and the epithelial-to-mesenchymal transition by suppressing the TGF-*β*1 signaling pathway [28, 29].

The molecular mechanism of Chinese herbal medicine in the treatment of PF has recently been predicted and verified using pharmacological networks. Jinyin granules are TCM compounds with detoxification, analgesic, and anti-inflammatory effects. They might alleviate PF progression through several signal pathways, such as Janus kinase 2/signal transducers and activators of transcription and the mammalian nuclear factor-*κ*B signaling pathway [30]. The Qimai feiluoping decoction is another TCM compound for treating PF associated with COVID-19 by supplementing Qi, nourishing Yin, and activating blood circulation. Pharmacological networks have predicted that Qimai feiluoping decoction exerts anti-PF effects *via* regulation of the epithelial-mesenchymal transition, extracellular matrix degradation, and TGF-*β* signaling pathway, and this has been verified *in vitro* [31]. Pharmacological networks have also found that Chinese herbs such as Curcuma Radix [32], Houttuynia cordata [33], Schisandra [34], and Astragalus can regulate PF *via* the TGF-*β*, PI3K/Akt, MAPK, and STAT3 signaling pathways. Astragalus is the most popular Chinese herb for supplementing Qi and is the main ingredient of the representative Buyang Huanwu decoction that also activates blood circulation. Pharmacological networks have shown that the IL-17, EGFR, and HIF-1 signaling pathways are the most closely associated with the mechanism of Astragalus in the treatment of PF and that PTGS2, VEGFA, MMP-9, STAT3, and EGFR are hub targets [35].

The main medicinal substances of Astragalus are astragaloside IV, Astragalus polysaccharide, and Astragalus flavonoids. Astragaloside IV reduces PF induced by BLM [36] or silica [12] through the TGF-*β*1/Smad3 signaling pathway. Its mechanism of action is associated with the inhibition of inflammatory factor expression and the modulated conversion of damaged alveolar cells to myofibroblasts in PF [37], as well as extracellular matrix deposition [38]. Astragalus polysaccharides inhibit the NF-*κ*B signaling pathway and the epithelial-mesenchymal transformation to reduce PF [13]. Astragali Radix extract injection contains astragaloside IV, Astragalus polysaccharides, and other chemical components. It is approved in China for treating viral myocarditis, cardiac insufficiency, hepatitis, and other diseases related to a weakness of righteous Qi. The scope of AI application has recently expanded, especially to diseases associated with fibrosis, such as diabetic nephropathy [39]. Although AI attenuates alveolitis and fibrosis scores in BLM rats, few studies have focused on the function of AI in PF [40].

Transplantation with MSCs is a new approach to PF treatment. These cells in animal models of bleomycin-induced PF can improve the extent of collagen deposition in the lungs, reduce TGF-*β* levels, decrease neutrophil counts in bronchoalveolar lavage fluid, and improve survival [41]. Clinical trials have shown that intravenous MSCs are effective and safe for treating patients with severe IPF, improving lung function and fibrosis scores under CT, and increasing the 6-min walk distance. The most common source of MSCs in clinical trials of MSCs as IPF treatment is the bone marrow [15]. After transplantation, BMSCs can migrate to damaged lung tissues, modulate immune cell function, reduce local inflammation, and inhibit fibrosis through various pathways such as paracrine secretion. Astragaloside IV [42] and astragaloside polysaccharides both promote the proliferation and differentiation of BMSCs after transplantation [43]. The present study found that the therapeutic effects of AI with and without BMSCs in BLM rats are due to the modulating effects of active Astragalus polysaccharides on BMSCs.

Patients with PF present with progressively worsening dyspnea associated with progressive interstitial fibrosis leading to persistently impaired lung function. The alveolar septa and capillary walls thicken in fibrotic lung tissues, causing a reduced ventilation-perfusion ratio and impaired oxygen diffusion. Fibrotic tissues have increased elastic recoil and reduced lung expansibility, resulting in a reduction in total lung volume [44]. Thus, tidal volume, FVC, and lung compliance are always reduced in patients with PF [45]. Patients with advanced PF often develop hypoxemia and require continuous supplemental oxygen therapy. Our findings showed that the model rats had lower FVC and lung compliance than the sham group and that AI with or without BMSCs improved the impaired lung function in BLM rats. Excessive extracellular matrix deposition is one cause of the reduced lung function in PF, and collagen is a major component of the extracellular matrix. We also found that AI with BMSCs attenuated the expression of collagen I and collagen III in the lung tissues of BLM rats.

The pathogenesis of PF involves various immune and inflammatory factors, among which TGF-*β* is an essential promoter of PF development. It has the subtypes TGF-*β*1, TGF-*β*2, and TGF-*β*3, of which TGF-*β*1 is most closely associated with fibrotic disease [46]. On the one hand, TGF-*β*1 regulates the Smad pathway and recruits circulating fibroblasts to the lungs while promoting epithelial- and endothelial-mesenchymal transitions, intrapulmonary fibroblast proliferation, and extracellular matrix deposition [47]. On the other hand, TGF-*β*1 can induce macrophage recruitment, activate signaling pathways such as JNK, p38, and ERK, produce various inflammatory factors such as IL-1*β*, and aggravate inflammatory injury. The present study found a significantly increased TGF-*β*1 expression level in BLM rats and that AI and BMSCs inhibited it.

Matrix metalloproteinases are enzymes that degrade the extracellular matrix and can activate TGF-*β*1. Their balance is closely associated with extracellular matrix deposition, lung tissue remodeling, and immune inflammation [48]. The regulation of MMPs is significantly imbalanced in BLM animal models, in which MMP expression level is elevated during the early inflammatory phase and relatively decreased during the late fibrotic phase, along with increased expression levels of inhibitory TIMPs and decelerated collagenolysis in lung tissues, all of which promote the formation and development of PF [49]. Although the expression levels of MMPs were reduced in BLM rats during the fibrotic repair phase compared with the inflammatory phase, they were still higher than those in normal control rats. During the fibrotic repair phase, MMPs are expressed mainly by type II alveolar epithelial cells surrounding fibrotic lesions, thus promoting tissue repair [50]. The regulation of MMPs is one pathway to improving PF and an important mechanism for treating PF with BMSCs. We showed that AI and BMSCs inhibited the increased expression levels of MMP-1, MMP-2, MMP-3, MMP-9, and their inhibitor TIMP-1 in BLM rats, which agreed with previous findings [51]. However, AI + BMSC increased serum levels of MMP-2, MMP-3, MMP-9, and TIMP-1 and inhibited collagen I and collagen III mRNA expression in lung tissues. The balance between MMPs and TIMPs is an important mechanism regulating the deposition of the extracellular matrix. The balance between low and high expression of MMPs and TIMPs influences PF, which requires future investigation.

The processes through which BMSCs are captured in the pulmonary vasculature after intravenous transplantation and migrate from the endothelium to the site of damage are collectively known as homing; this is a crucial component in determining the repair role of these cells. Stem cell homing is closely associated with chemokines and their receptors, especially the CXCL12/CXCR4 signaling axis [52]. Chemokine CXCL12 (a.k.a. matrix-derived factor 1*α*) is a specific chemokine attractant protein, and CXCR4 is a specific receptor for CXCL12 and BMSCs. The CXCL12/CXCR4 signal axis can regulate the chemotaxis, homing, proliferation, and survival of BMSCs [53]. We also found that CXCL12, CXCR4, and CD90 are expressed in bone marrow mesenchymal stem cells. The expression of CXCL12 and CD90 was significantly more abundant in the AI + BMSC than in the BLM, AI, and BMSC groups, suggesting that Astragalus increases the directional migration of BMSCs to damaged lung tissues by promoting CXCL12 expression.

Although this study showed that AI alone or in combination with BMSCs reduced TGF-*β*1 expression level, attenuated collagen deposition in the lungs, and elevated FVC and CYDN in BLM rats, it has many limitations. The mechanism of action of the drug in alleviating PF in BLM rats should be explored in depth. Changes in the CXCL12/CXCR4 signal axis and BMSC surface marker CD90, which regulate the directional migration of BMSCs, should be assessed more accurately at the protein level. The modulation of inflammatory factors is an essential mechanism of PF alleviation by Astragalus and its active ingredients. In fact, the present study was also designed to examine inflammatory factors such as IL-1*β*, IL-6, and TNF-*α* in serum. However, the levels of these inflammatory factors did not significantly differ. We investigated the effects of AI and BMSCs only *in vivo*. Therefore, studies *in vitro* are needed to investigate the mechanisms of drug action in more detail.

## 5. Conclusions

Astragali Radix extract injection combined with BMSCs alleviated collagen deposition in the BLM-affected rat lungs and improved their function. This effect may have been associated with the regulation of MMP, TGF-*β*1, TIMP-1, and the CXCL12/CXCR4 signaling axis.

## Figures and Tables

**Figure 1:** Scheme of the study design.

**Figure 2:** Surface expression of antigen CD90 on BMSCs from SD rats (magnification, 200x). BMSCs, bone marrow mesenchymal stem cells; CD90, cluster of differentiation 90; SD, Sprague-Dawley.

**Figure 3:** Lung function and pathological sections. (a, b) Lung function changes. (c–h) HE-stained sections (magnification, 100x). (i–o) Collagen-stained blue with Masson trichrome staining (magnification, 100x). ^*∗∗*^*P* < 0.01, ^*∗∗∗*^*P* < 0.001, and ^*∗∗∗∗*^*P* < 0.0001 vs. BLM. BLM, bleomycin; HE, hematoxylin, and eosin.

**Figure 4:** Expression of TGF-*β*1 and matrix metalloproteinases and matrix metalloproteinase inhibitors. (a) TGF-*β*1, (b) MMP-1, (c) MMP-2, (d) MMP-3, (e) MMP-9, (f) TIMP-1, (g) collagen I, and (h) collagen III. ^*∗*^*P* < 0.05, ^*∗∗*^*P* < 0.01, ^*∗∗∗*^*P* < 0.001, and ^*∗∗∗∗*^*P* < 0.0001 vs. BLM. ^##^*P* < 0.01, ^###^*P* < 0.001, and ^####^*P* < 0.0001 vs. BMSC or AI. BLM, bleomycin; AI, Astragali Radix extract injection; BMSC, bone marrow mesenchymal stem cells; MMP, matrix metalloproteinases; TIMP, tissue inhibitor matrix metalloproteinase.

**Figure 5:** Effects of AI and BMSCs on (a) CXCL12, (b) CXCR4, and (c) CD90 expression. ^*∗*^*P* < 0.05, ^*∗∗*^*P* < 0.01, ^*∗∗∗*^*P* < 0.001, and ^*∗∗∗∗*^*P* < 0.0001 vs. BLM. ^##^*P* < 0.01, ^###^*P* < 0.001, and ^####^*P* < 0.0001 vs. BMSC or AI. BLM, bleomycin; AI, Astragali Radix extract injection; BMSCs, bone marrow mesenchymal stem cells; CD90, cluster of differentiation; CXCL12, C-X-C motif chemokine ligand 12; CXCR4, C-X-C Chemokine Receptor 4.

**Table 1:** Primer sequences.

Gene name	Primer sequences (5′-3′)
*β*-Actin	Forward: TGTCACCAACTGGGACGATA
	Reverse: GGGGTGTTGAAGGTCTCAAA

CXCR4	Forward: AAGCAAGGATGTGAGTTCGAGAGC
	Reverse: CCGAGGAAGGCGTAGAGGATGG

CD90	Forward: ACACATACCGCTCCCGAACCAAC
	Reverse: GGGCCCCACCAGTCACAGG

Collagen I	Forward: AGTCTCAAGATGGTGGCCGT
	Reverse: CAATCTGCTGGCTCAGGCTC

Collagen III	Forward: AGTCGGAGGAATGGGTGGCTATC
	Reverse: CAGGAGATCCAGGATGTCCAGAGG

## Data Availability

The original data in this study are included in this article.
